# Circular RNAs and their roles in head and neck cancers

**DOI:** 10.1186/s12943-019-1003-5

**Published:** 2019-03-21

**Authors:** Yang Guo, Jiechao Yang, Qiang Huang, Chiyao Hsueh, Juan Zheng, Chunping Wu, Hui Chen, Liang Zhou

**Affiliations:** Department of Otorhinolaryngology Head and Neck Surgery, Shanghai Key Clinical Disciplines of Otorhinolaryngology, Eye & ENT Hospital of Fudan University, Shanghai, People’s Republic of China

**Keywords:** Circular RNA, Biogenesis, Characteristics, Head and neck cancer, Sponge function, Biomarker

## Abstract

Circular RNAs are abundant endogenous non-coding RNA with no 5′ cap and 3′ polyadenylation tail that modify liner mRNAs and have no terminal structures. Our knowledge of the biogenesis of circular RNAs has been expanded, and circular RNAs were shown to be key regulators of various diseases, especially cancers. Head and neck cancers are the sixth most popular cancers worldwide, and the overall survival rates remain unsatisfactory. Recent studies have indicated that circular RNAs are involved in the tumorigenesis, progression, invasion and chemosensitivity of head and neck cancers and that some circular RNAs could serve as diagnostic and prognostic biomarkers. In this study, we summarize research advances in the regulation of circular RNA biogenesis, their characteristics and functions, the involvement of circular RNAs in the pathophysiology of head and neck cancers and their potential clinical utilization, as well as the likely directions of future studies.

## Background

Head and neck cancers (HNCs) are the sixth most popular cancer worldwide [1, 2]. Over 500,000 new cases are diagnosed and approximately 300,000 deaths occur each year [3]. Among the malignancies located at various subsites in the head and neck, head and neck squamous cell carcinomas (HNSCCs) accounted for the vast majority of HNCs [4]. Despite the development of various therapeutic methods, including surgery, chemotherapy, radiation therapy, induction chemotherapy and immunotherapy [5], the overall survival rates of HNCs have not been improved in recent decades. Thus, elucidation of the underlying molecular mechanism is needed to improve therapeutic efficacy. 

Extensive research efforts on the carcinogenesis, development and effective therapeutic methods of HNCs, in which non-coding RNAs (ncRNAs), such as microRNAs (miRNAs) and long ncRNAs (lncRNAs), were inevitably involved, have been conducted [6, 7]. Researchers suggested that ncRNAs comprise most of the human transcriptome, while protein-coding genes accounted for only a tiny sliver, less than 2%, of the total genome [8, 9]. Recently, with the rapid development of novel bioinformatics approaches and next-generation sequencing (NGS), particularly the RNA-seq technique, a subclass of ncRNAs named circular RNAs (circRNAs) has attracted increased attention from global researchers [10]. CircRNAs were first found approximately 40 years ago in viroids and RNA viruses [11, 12] and were then found soon after in eukaryote cells [13]. Compared to miRNAs and lncRNAs, circRNAs are much more stable due to the circular structure. Many biological and physical processes have been demonstrated to be regulated and influenced by various circRNAs, especially processes in cancers.

In the emerging landscape of circRNAs, circHIPK3 is one of the most thoroughly explored circRNAs. As a typical competing endogenous RNA (ceRNA), circHIPK3 was shown to have up to 18 miRNA response elements (MREs) for 9 miRNAs [14]. CircHIPK3 could abrogate the functions of target miRNAs by binding them. CircHIPK3 is involved in various biological and physiological processes, such as diabetic retinopathy [15], age-related cataracts [16], diabetes [17] and diverse types of cancers [14, 18–20]. CircHIPK3 plays oncogenic roles through binding to miR-124 in hepatocellular carcinoma [21] and gallbladder cancer [22]. By sponging miR-7 and miR-654, respectively, circHIPK3 could promote the progression of colorectal cancer [23] and glioma [24]. However, circHIPK3 could suppress the migration, invasion, and angiogenesis of bladder cancer by abolishing the effect of miR-558 [18]. Similarly, circHIPK3 also serves as an antioncogenic circRNA in osteosarcoma [25].

The “sponge” mechanism is the most popular function of circRNAs [26, 27], and many studies on the “sponge” functions of circRNAs in cancer have been undertaken [18, 28–38]. Additionally, circRNAs could be secreted into blood, saliva [39] and even exosomes [33], which play important roles in the tumor microenvironment.

Meanwhile, knowledge regarding the functions and mechanisms of circRNAs in HNCs has been accumulated. Elucidation of the characteristics and functions of circRNAs at the genetic and molecular levels is urgently needed for the development of novel therapies and precision medicines for HNCs [40]. In this paper, we discuss the research advances in circRNAs and summarize the roles of circRNAs and their likely clinical application value in HNCs. The innovations of our manuscript mainly lie in the systemic depiction of the RNA binding proteins (RBPs) involved in the biogenesis of circRNAs, the protein reservoir function of circRNAs, the interactions between RBPs and circRNAs in physiological and pathophysiological conditions and the potential biomarkers for HNCs.

## Classification of circRNAs

Based on the biogenesis of circRNAs in human cells, these molecules could be divided into three main kinds: exonic circRNAs (ecircRNAs) and intronic circRNAs (ciRNAs) generated from the exons and introns in the pre-mRNAs, respectively, and exon-intron circRNAs (EIciRNAs) consisting of both exons and introns from the pre-mRNAs (Fig. 1) [41]. EcircRNAs are formed by the back-splicing that attaches the downstream 5′ splice donor to the upstream 3′ splice acceptor. If the introns between the 5′ splice donor and the 3′ splice acceptor are not removed by canonical splicing, the resultant circRNAs are regarded as EIciRNAs. The ciRNAs are produced from intronic regions after the release of the 3′ exon by forming a branchpoint 2′–5′ linkage between the terminal 2′-OH group of the intron and the 5′ splice site. Then, the 3′ tail is degraded, forming the final ciRNA [42, 43]. Through a 7-nt GU-rich motif near the 5′ splice site and an 11-nt C-rich motif at the branchpoint site, the mature ciRNAs escape from further debranching and degrading [43, 44].

**Fig. 1:** The formation and classification of circRNAs. Canonical splicing produces liner mRNAs (**a**) while back-splicing generates circRNAs (**b**). **b**. CircRNAs were usually categorized into ecircRNAs, ciRNAs and EIciRNAs depending on their components, which were derived from exons and introns, and both of them in pre-mRNAs, respectively. Different ecircRNAs could be generated from one pre-mRNA via alternative splicing. The red segment and yellow segment between Exon 4 and Exon 5 represented a 7-nt GU-rich motif near the 5′ splice site and an 11-nt C-rich motif at the branchpoint site, respectively, which promoted the generation of ciRNAs

In addition to the circRNAs mentioned above, one special type of circRNA, fusion circRNAs (f-circRNAs), generated from fusion genes formed by cancer-associated chromosomal translocations, has recently been described [45]. F-circRNAs consist of exons from otherwise separated genes that were fused by aberrant chromosomal rearrangements [45, 46].

## Mechanisms of ecircRNA biogenesis and RBP regulation of ecircRNA biogenesis

The vast majority of circRNAs are ecircRNAs, while the numbers of ciRNAs and EIciRNAs are low [18, 41, 47–49]. Thus, we focused on the regulation of ecircRNA biogenesis here.

Generally, three models have been developed to illustrate the mechanisms of ecircRNA synthesis. The circularization of ecircRNAs is usually stimulated by the complementary sequences of the introns in the pre-mRNAs, which is known as intron pairing-driven circularization [41, 50, 51]. The pairing across complementary sequences in the flanking introns of the circularized exons brought the splicing sites into proximity, facilitating the circularization of the intervening exons (Fig. 2b). With expression plasmid mutagenesis, Liang et al. confirmed that even introns as short as 30–40 nts comprising repeat inverted sequences (such as *Alu* elements) were able to circularize the intervening exons in human cells [52]. Additionally, this model was refined by the alternative splicing theory, which could explain the different ecircRNAs generated from one parental gene (Fig. 1b) [47, 51, 53].

**Fig. 2:** Three models for the biogenesis of ecircRNAs. **a**. Lariat-driven circularization, also known as the exon-skipping model. The remaining exons in the pre-mRNAs were allocated into the concomitant linear mRNAs. **b**. Intronic base pairing-driven circularization. The pairing across complement sequences in the flanking introns brought the splicing sites into proximity, facilitating the circularization of intervening exons. **c**. RBP-driven circularization. The interactions of RBPs binding to the flanking introns serve as a bridge to bring the introns into proximity, promoting the process of circularization. **d**, **e**. Some RBPs could bind to the intronic dsRNA to regulate the biogenesis of ecircRNAs. While some RBPs (such as NF90/NF110) stabilize the dsRNAs to promote the generation of ecircRNAs (**d**), some RBPs (such as DHX9 and ADAR1) destroy the stability of dsRNAs to suppress the generation of ecircRNAs (**e**)

In addition to the above intron pairing-driven circularization, ecircRNAs could be developed through one other model called lariat-driven circularization, namely, the exon-skipping model [41, 54–58]. During the formation of linear RNA from pre-mRNA, the splicing sites of skipped exons are joined through the construction of a lariat. After the introns in the lariat are removed, ecircRNAs are produced (Fig. 2a).

In addition, over one hundred RNA-binding proteins (RBPs) were proposed to be involved in the regulation of ecircRNA biogenesis [59], and the regulatory mechanisms of some RBPs, such as quaking (QKI), muscleblind (Mbl), nuclear factor 90/110 (NF90/NF110), adenosine deaminases that act on RNA 1 (ADAR1) and DExH-box helicase 9 (DHX9), have been illuminated (Table 1) [59–64]. Some RBPs could bind to the flanking introns of single-stranded RNAs to bring them into vicinity, thus promoting the generation of ecircRNAs (Fig. 2c). By binding to intronic QKI binding motifs in the vicinity of the circRNA-forming splice sites, the upregulated QKI promotes the generation of ecircRNAs during epithelial-mesenchymal transition (EMT). In addition, the appropriate insertion of QKI binding sites into the adjacent introns of exons would facilitate the formation of ecircRNAs instead of canonically formed mRNAs [62]. A positive correlation was found between the expression levels of QKI and the overall expression of ecircRNAs [62, 65]. Analogously, overexpressed MBL bound to MBL binding sites in introns flanking the second exon, the circRNA-forming exon, of its parental gene MBL to induce circularization, and this mechanism was conserved from *Drosophila* to human [60]*.* FUS also mainly binds to the proximal intron regions of the back-splicing junctions to regulate ecircRNA biogenesis [66]. However, while MBL promoted the biogenesis of circMbl at the expense of canonical co-transcriptional linear splicing, which produced corresponding linear RNA, FUS was shown to regulate the generation of ecircRNAs post-transcriptionally independent of the expression levels of the cognate linear RNAs [66]. Likewise, heterogeneous nuclear ribonucleoprotein L (HNRNPL) participated in the regulation of ecircRNA formation with a similar mechanism to FUS [67]. RNA-binding motif protein 20 (RBM20) is a splicing factor implicated in dilated cardiomyopathy (DCM), which regulates the alternative splicing within the I-band of the titin gene [68]. Khan et al. showed that by providing the substrate for the generation of ecircRNAs, RBM20 could accelerate the generation of ecircRNAs from the I-band of the titin gene through excluding specific exons from the pre-mRNA [69]. In addition, the RNA splicing proteins heterogeneous nuclear ribonucleoprotein (hnRNPs) and serine–arginine (SR) act in combination with base pairing introns to coordinate the production of ecircRNAs [70]. However, some RBPs function by interacting with double-stranded RNA (dsRNA) to influence the biogenesis of ecircRNAs. For instance, the dsRNA-editing enzyme ADAR1 suppresses the expression of the ecircRNAs by “melting” the paired intronic sequences through A-to-I editing. In addition, knockdown of ADAR1 specifically upregulated ecircRNA expression [61, 64]. Similarly, Aktaş et al. showed that knockdown of the RNA helicase DHX9, which targets long dsRNA formed by base pairing *Alu* elements, resulted in increased ecircRNA-producing genes and levels of ecircRNAs [71]. There was a synergistic effect between DHX9 and ADAR1 on the regulation of ecircRNA generation (Fig. 2e) [71]. In the nucleus, NF90/NF110 preferentially binds to the flanking introns of circularized exons rather than other introns. NF90/NF110 stabilize the double-stranded intronic RNA pairs and juxtapose the ecircRNA-forming exons, facilitating the biogenesis of ecircRNAs (Fig. 2d) [59].

**Table 1:** The RNA binding proteins (RBPs) involved in the regulation of ecircRNA biogenesis

Proteins	Target RNA	Target sites	Functions	Possible mechanism	Features	Reference
QKI	Single strand RNA	QKI binding sites in flanking introns of circRNA-forming exon	Positive	Bringing the flanking introns into vicinity to facilitate the circularization	Inserting QKI binding sites into the adjacent introns of exons appropriately would facilitate the formation of circRNAs instead of mRNAs formed canonically	[62]
MBL	Single strand RNA	MBL binding sites in flanking introns of circRNA-forming exon	Positive	Bringing the flanking introns into vicinity to facilitate the circularization	Generation of circRNAs compete with canonical cotranscriptional linear splicing; Mbl promote the circMbl at the expense of linear splicing; efficient MBL-induced circularization depends more on the binding of MBL to both introns simultaneously than on the total number of MBL binding sites	[60]
FUS	Single strand RNA	FUS binging sites in introns flanking the back-splicing junctions	Positive/negative	Through protein-protein and RNA-protein complexes	FUS regulate the biogenesis of circRNA independent of the cognate linear RNA; nuclear located circRNAs facilitated by FUS were consisted of entirely of exonic sequences	[66]
HNRNPL	Single strand RNA	HNRNPL binding sites in flanking introns of circRNA-forming exon	Positive/negative	HNRNPL binding on both sides of flanking introns presented stronger promoting effect on circRNA formation than on one side; more binding sites correlated with elevated chances to form circRNA	HNRNPL regulate the biogenesis of circRNA independent of the cognate linear RNA; among the circRNAs regulated by HNRNPL, upregulated circRNAs were related to HNRNPL binding more intensely than downregulated circRNAs if the binding occured at flanking introns or within the circRNAs	[67]
RBM20	Single strand RNA	RBM20-binding sites in the introns flanking the titin circRNAs	Positive	Provide the substrate to form RBM20-dependent circRNAs post-transcriptionally by excluding specific exons from the pre-mRNA	As RBM20 is the splicing factor responsible for alternative splicing within the I-band of the titin gene, it is crucial for the formation of circRNAs originated from the I-band (ie, Ig and PEVK domain)	[69]
hnRNPs and SR	Single strand RNA	Specific binding sites in flanking introns	Positive/negative	Probably through aiding or blocking spliceosome assembly	The effects of hnRNPs, and SR proteins were coordinated with the effect of intronic repeats in a combinatorial manner	[70]
ADAR1	Double strand RNA	Basepaired dsRNA proximal to the splice sites of circularized exons	Negative	Destroy the paired intronic sequences through A-to-I editing	CircRNAs could be upregualted independently of the expression level of the linear mRNA through ADAR1 depletion	[61, 64]
DHX9	Double strand RNA	Long dsRNA formed by base pairing *Alu* elements	Negative	Might break the paired intronic sequences through resolving inverted-repeat *Alu* elements	DHX9 exists a synergistic effect with ADAR on circRNA production	[71]
NF90/NF110	Double strand RNA	Transient dsRNAs duplexes formed by circRNA-flanking *cis* complementary sequences	Positive	Stabilizing flanking intronic RNA pairs to promote circRNA processing	NF90 selectively bound to flanking introns of circularized exons and NF90 preferred to bind clusters of A-rich or U-rich sequences, most of which located *Alus* in introns	[59]

Notably, the RBPs that regulate ecircRNA biogenesis also displayed evolutionary conservation, in addition to the conserved expressed ecircRNAs across species described below. For example, exogenous expression of *Drosophila* MBL could stimulate the generation of endogenous circMbl in human cells despite the differently dominant splicing mechanisms between flies and mammals [60]. Likewise, the regulatory effects of FUS [66] and ADAR1 activity on the production of ecircRNAs were also suggested to be conserved from mice or flies to humans [64].

## Other factors affecting the biogenesis of ecircRNAs

Moreover, the expression of ecircRNAs could be influenced by the efficiency of linear splicing in the host genes. If the elongation capacity of RNA polymerase II was abrogated, co-transcriptional splicing efficiency would be increased, which resulted in decreased ecircRNA expression [60, 72]. When the core spliceosomal components were depleted, which decreased the canonical mRNA splicing rate or RNA polymerase II termination efficiency, the biogenesis of ecircRNAs could be increased [73].

Studies have suggested that other factors, such as the length of the circularized exons and flanking introns of the circularized exons, as well as transcription factors, could also affect the biogenesis of ecircRNAs [41, 47, 55, 58, 70, 74–76]. Recently, the EMT–inducing transcription factor Twist1, which targets the promoter of Cul2, was proved to increase the expression of circCul2 (circRNA-10720), specifically while repressing cognate mRNA [77]. For f-circular RNAs, other mechanisms in addition to back-splicing might be involved [46]. Although the regulation of ecircRNAs has been extensively studied, further studies are still needed to decipher the underlying mechanisms.

## Characteristics of circRNAs

### Stability

CircRNAs are much more stable than mRNAs because of the closed loop structure. The absence of free terminals endows them with resistance to exonucleases. The half-lives of circRNAs are approximately 24–48 h, while those of liner RNAs are only approximately 8–9 h [14, 44, 78].

### Abundance

CircRNA expression is widespread in different species from plants to animals, such as *Arabidopsis thaliana* [79], rice [49], *Caenorhabditis elegans* [80], mice [81] and humans [64]. In humans, circRNAs are generally expressed in the vast majority of tissues and are especially abundant in the brain [64, 82, 83]. This abundance may have resulted from the accumulation of stable circular RNAs that are exonuclease-resistant and the high speed of biosynthesis [41, 64]. CircRNAs were found to be the predominant RNA isoforms for hundreds of human genes [74], of which the expression levels could be up to 10-fold~ 20-fold of the levels of their linear isoforms [41, 64, 84].

### Conservation

Many circRNAs were proven to be highly conserved between human brain and mouse brain, and some of the conserved circRNAs were even identified in fly head [64]. Recently, Dong et al. demonstrated that approximately 15,000 circRNAs were conserved between humans and mice, accounting for 40% of the total circRNAs in mice [85], which was similar to the proportion of 4522 out of 15,849 reported by Rybak-Wolf et al. [64]. Moreover, conserved circRNAs were present at higher levels than non-conserved circRNAs [64, 85, 86].

### Specificity

Although several circRNAs were proven to be conserved across species, the majority of circRNAs showed species-specific expression [85]. The total circRNAs detected tended to increase with the evolution of species, which was also true for the circRNAs generated from orthologous genes [85].

In addition, circRNA expression was usually cell-specific, tissue-specific and developmental stage-specific [49, 75, 76, 82–84, 86–88], indicating that the balance between biogenesis and turnover of circRNAs was under strict control.

Moreover, circRNA expression was disease-specific. The most representative circRNAs were the f-circRNAs previously shown to result from disease-specific chromosomal translocations [45, 46, 89].

### Distinct localization

EcircRNAs are predominantly localized in the cytoplasm [41], while ciRNAs and ElciRNAs were preferred localized in the nucleus [43, 90]. This finding may be related to the distinct molecular roles of various kinds of circRNAs in cells. An increasing number of studies have indicated that ecircRNAs in the cytoplasm act as miRNA sponges through MREs, while nuclear ElciRNAs regulate gene transcription as scaffolds of proteins in the nucleus [14, 22, 90].

However, there are exceptions. Recently, the nuclear circRNAs promoted by FUS were shown to consist of complete exons [66], and circSEP3, which was generated from exon 6 of SEPALLATA3 (SEP3) in *Arabidopsis*, was also retained in the nucleus to regulate splicing of its cognate linear mRNA [91].

## Functions of circRNAs

### Functions as miRNA sponges

Taking the abundance and cell-, tissue-, development-, and disease-specificity of circRNAs into account, researchers supposed that circRNAs play essential roles in various biological functions [42, 56, 92]. One of the most widely studied functions of circRNAs is their roles as miRNA sponges in the cytoplasm [26, 93]. The most representative circRNA is Cdr1as (antisense to the cerebellar degeneration-related protein 1 transcript), which has more than 70 MREs for miR-7 [93]. By targeting different miRNAs and downstream mRNAs, circRNAs are involved in the pathological mechanism of diverse diseases, including neurological diseases [94, 95], cardiovascular disease [96, 97], cartilage degradation [98], diabetes [99], pulmonary fibrosis [100, 101], and in particular various cancers [18, 29, 102, 103]. Additionally, circRNAs store and transport miRNAs through binding miRNAs to the MREs, and the sponged miRNAs could be released to function under special conditions [56, 93, 104].

### Protein reservoirs or interactions with RBPs

Similar to the absorption of miRNAs, circRNAs sponge proteins and serve as reservoirs (Table 2) [34, 105]. CircMbl binds to MBL to terminate its enhancement of the generation of circMbl, constructing a feedback loop regulating the balance of circMbl and its cognate linear mRNA [60]. Another example is the immune factors NF90/NF110, which could be transported to the cytoplasm and detached from circRNAs to bind to viral mRNAs inhibiting viral replication upon viral infection [59]. Similarly, c-myc is translocated to the nucleus and stabilized by binding to circAmotl1, participating in tumorigenesis [34]. In addition, circDNMT1 could bind to p53 and AUF1 to facilitate their nuclear translocation, accelerating breast cancer progression via activating autophagy [106]. Furthermore, circAmotl1 could promote the nuclear translocation of STAT3 to stimulate wound healing [105]. Additionally, circPABPN1 binds to HuR to compete with the binding of HuR to PABPN1 mRNA [107].

**Table 2:** The circRNAs could sponge proteins and circRNAs capable of interacting with RBPs

CircRNAs	Functions	Proteins	Possible mechanism involved in physiological process and pathophysiologic	Reference
circMbl	Protein reservoirs	Mbl	CircMbl could absorb MBL to terminate its promotion effect on the generation of circMbl, constructing a feedback loop regulating the balance of circMbl and its cognate linear mRNA	[60]
circRNP	Protein reservoirs	NF90/NF110	During the viral infection, NF90/NF110 was exported from nucleus by circRNPs and then released to bind to viral mRNAs for antiviral immune response	[59]
circAmotl1	Protein reservoirs	c-myc	Circ-Amotl1 induced nuclear translocation of c-myc, promoting c-myc stability and upregulating c-myc targets to accelerate tumorigenesis	[34]
circAmotl1	Protein reservoirs	Stat3	By binding to Stat3, circAmotl1 lead the nuclear translocation of Stat3, accelerating wound healing process via modulating Dnmt3a and miR-17 function	[105]
circPABPN1	Protein reservoirs	HuR	CircPABPN1 could suppress the translation of cognate mPABPN1 by binding to HuR, an RBP that could promote the translation of PABPN1 mRNA	[107]
circDNMT1	Protein reservoirs	p53 and AUF1	Both p53 and AUF1 undergo nuclear translocation through interacting with circ-Dnmt1. Nuclear translocated p53 promoted cellular autophagy while AUF1 nuclear translocation resulted in increased Dnmt1 translation	[106]
circFoxo3	Interact with RBPs	p21 and CDK2	CircFoxo3 repressed cell cycle in G1 phase by binding to the cell cycle proteins CDK2 and p21, forming a ternary complex as well as circFoxo3-CDK2 complex and circFoxo3-p21 complex	[110]
circFoxo3	Interact with RBPs	ID-1, E2F1, FAK, and HIF1a	CircFoxo3 was mainly located in the cytoplasm interacting with anti-senescent protein ID-1 and E2F1, the anti-stress proteins FAK and HIF1a retained in cytoplasm to abrogate their anti-senescent and anti-stress functions	[111]
circFoxo3	Interact with RBPs	p53 and MDM2	By binding to MDM2 and p53, circFoxo3 facilitated MDM2-induced p53 ubiquitination and subsequent degradation while freeing Foxo3 from being ubiquitinated, thus improved the level of PUMA which induced cell apoptosis	[112]
CircCcnb1	Interact with RBPs	H2AX and Bclaf1; H2AX and p53	In the conditions of p53 was mutant, circ-Ccnb1 could form a complex with H2AX and Bclaf1 to decrease the ability of proliferation and survival but increase the apoptosis; in the conditions of wild-type p53, circCcnb1 bind to H2AX and wild-type p53, avoiding induction of cell death	[113]

CircRNAs also bind to RBPs participating in various physiological processes (Table 2) [108, 109]. By forming ternary complexes with p21 and CDK2, circFoxo3 plays an anti-oncogenic role by blocking the cell cycle [110]. Additionally, circFoxo3 could lead to cellular senescence via binding to anti-senescent proteins and anti-stress proteins [111]. Furthermore, circFoxo3 could bind both p53 and MDM2, reinforcing the poly-ubiquitination function of MDM2 on p53, thus rescuing Foxo3 from degradation by MDM2 and inducing apoptosis [112]. CircCcnb1 interacts with H2AX and Bclaf1, forming a complex in p53 mutant cells to induce the death of cancer cells; however, by binding to H2AX and wild-type p53, circCcnb1 avoids the induction of cell death [113].

### Regulation of transcription and splicing

EcircRNAs showed different regulatory patterns on the transcription and splicing of their parental genes. First, ecircRNAs could regulate the linear splicing of their parental genes by competing for splice sites. While the expression of circMbl was upregulated by MBL overexpression, the expression of linear MBL was correspondingly decreased [60]. Second, the circularized exons forming ecircRNAs through exon-skipping were absent in the processed mRNAs. In other words, ecircRNA formation was associated with alternative splicing in the linear mRNAs [51, 55, 114]. In addition, the expression of host genes and other genes could be regulated by circRNAs through sponging various miRNAs targeting different genes [115–117]. Furthermore, circRNAs could bind to proteins to regulate the transcription of their locus genes. For example, EIci-EIF3J and EIci-PAIP2 could *in cis* promote the transcription of their parental genes through binding to U1 small nuclear ribonucleoprotein (snRNP), forming EIciRNA–U1 complexes that further interact with polymerase II at the gene promoter regions [90]. In addition, ciRNAs such as ci-ankrd52 and ci-sirt7 could regulate the transcription of their parental genes by interacting with polymerase II *in cis* [43].

### Translation and regulation of translation

As endogenous circRNAs were shown to be unable to recruit ribosomes [41, 83, 118], they were regarded as ncRNAs [56]. Recently, some endogenous circRNAs with open reading frames (ORFs) were found to be associated with translating ribosomes [119, 120]. Several circRNAs, such as circZNF609 and circMbl, could be translated in a cap-independent manner [119, 121]. Recently, circSHPRH [122] and circFBXW7 [123] were demonstrated to encode proteins suppressing the tumorigenesis of glioma. Furthermore, the N^6^-methyladenosine (m^6^A) residues in circRNAs were suggested to accelerate the cap-independent translations of circRNAs [120]. Bioinformation tools that could predict the protein coding potential of a certain circRNA, such as circRNADb [124] and CircPro [125], have been established.

In addition to being translational template for peptides, some circRNAs could regulate the translation of their cognate linear mRNAs. For example, the translation of PABPN1 was suppressed by circPABPN1 through competition for HuR, an RBP promoting translation [107].

### Biomarkers

Due to their stability and specificity, circRNAs are ideal biomarkers for various diseases [126–128], particularly cancers [33, 46, 129, 130].

Zhao et al. suggested that hsa_circ_0124644 in peripheral blood can be used as a diagnostic biomarker of coronary artery disease [126]. The upregulated circPVT1 in osteosarcoma patients was correlated with poor prognosis, and the diagnostic value of circPVT1 for osteosarcoma was higher than that of lactate dehydrogenase (LDH), one commonly used diagnostic biomarker in the clinic [37]. Similarly, hsa_circ_0000190 had better sensitivity and specificity for the diagnosis of gastric cancer than two classic biomarkers, carcinoembryonic antigen (CEA) and CA19–9 [31]. Furthermore, some circRNAs were enriched in exosomes, and circRNAs in serum exosomes could distinguish patients with tumors from healthy controls [33].

## CircRNAs in HNCs

### CircRNAs as biomarkers in HNCs

Ganci et al. reported that dysregulated miRNAs in tissues could predict the prognosis of HNCs [131–133]. The circulating miRNAs from blood, plasma or serum that could be promising biomarkers have been reviewed [134]. Similarly, potential lncRNA biomarkers for HNCs have been identified [135, 136]. Considering the stability, tissue-specificity and abundance of circRNAs [39, 129], these molecules are ideal potential biomarkers for precise treatment [40] of HNCs (Table 3).

**Table 3:** The potential circRNA biomarkers in HNCs

CircRNAs	Chromosome	Gene symbol	Primary sites of cancer	Expression change	Relationships with the clinical features	Number of patients	Cilinical samples	Clinical value	Reference
circPVT1	chr8	*PVT1*	HNSCC	Up	mut-p53, alcohol use	106	Tumor tissues	Poor overall survival (dependent on the TP53 mutations)	[137]
hsa_circ_0008309	chr2	*CUL3*	OSCC	Down	Pathological differentiation	45	Tumor tissues/Non-tumor tissues	Diagnosis biomarker (AUC = 0.764)	[138]
hsa_circ_001242	chr10	*TRDMT1*	OSCC	Down	Tumor size, T stage	40	Tumor tissues/Non-tumor tissues	Diagnosis biomarker (AUC = 0.784, Sensitivity = 0.725, Specificity = 0.775)	[139]
hsa_circ_0109291	chr19	*ZNF714*	OSCC	Up	TNM stage	51	Tumor tissues	Poor overall survival	[140]
hsa_circ_0001874	chr9	*BICD2*	OSCC	Up	TNM stage and tumor grade	178	Saliva from the OSCC patients and healthy controls	Early non-invasive diagnosis biomarker for OSCC in saliva (AUC = 0.863, Sensitivity = 0.744, Specificity = 0.902)	[144]
hsa_circ_0001971	chr7	*FAM126A*	OSCC	Up	TNM stage	178	Saliva from the OSCC patients and healthy controls	Early non-invasive diagnosis biomarker for OSCC in saliva (AUC = 0.845, Sensitivity = 0.756, Specificity = 0.878)	[144]
hsa_circ_0001874 + hsa_circ_0001971	–	–	OSCC	–	–	178	Saliva from the OSCC patients and healthy controls	Early non-invasive diagnosis biomarker for OSCC in saliva (AUC = 0.922, Sensitivity = 0.927, Specificity = 0.778)	[144]
hsa_circRNA_100855	–	–	LSCC	Up	T stage, lymph node metastasis, primary location, clinical stage	52	Tumor tissues/Non-tumor tissues	Diagnosis and prognosis biomarker*	[145]
hsa_circRNA_104912	–	–	LSCC	Down	T stage, differentiation, lymph node metastasis, clinical stage	52	Tumor tissues/Non-tumor tissues	Diagnosis and prognosis biomarker*	[145]
hsa_circ_0000284 (circHIPK3)	chr11	*HIPK3*	NPC	Up	Clinical stage, distant metastasis	63	Tumor tissues	Poor overall survival and distant metastasis-free survival rates	[146]
has_circ_0000285	chr11	*HIPK3*	NPC	Up	Tumor size, TNM stage, distant metastasis, tumor grade and lymph node metastasis	150	Serums and tumor tissues	Poor overall survival, poor radiosensitivity and serve as independent prognostic factors (HR = 3.03, *p* = 0.02)	[147]

Note: *HNSCC* head and neck squamous cell carcinoma, *OSCC* oral squamous cell carcinoma, *LSCC* laryngeal squamous cell carcinoma, *NPC* nasopharyngeal carcinoma, “-” means unannotated or not investigated in the paper, “*” means based on speculation but not validated clinically

CircPVT1 was upregulated in HNSCC tissues compared to matched normal tissues [137]. However, if HNSCC patients were divided into mut-p53 and wild-type groups, the expression levels of circPVT1 were only overexpressed in patients with TP53 mutations compared to those of non-tumor tissues. Furthermore, there was a significant correlation between circPVT1 and mut-p53, and the correlation between circPVT1 and alcohol use slightly missed the margin of significance. In addition, high circPVT1 predicted poor overall survival, which was dependent on the TP53 mutations [137].

High-throughput sequencing and qRT-PCR showed that hsa_circ_0008309 was downregulated in oral squamous cell carcinoma (OSCC) tissues compared with paired adjacent normal tissues (ANTs) [138]. Similarly, hsa_circ_001242 was downregulated in OSCC tissues and OSCC cell lines compared with ANTs and the human normal oral keratinocyte (hNOK) cell line [139]. The hsa_circ_0008309 expression level was significantly related to the tumor differentiation of OSCC, while hsa_circ_001242 expression levels were negatively associated with tumor size and T stage of OSCC. Receiver operating characteristic (ROC) curve analysis was performed to differentiate OSCC tissues from the ANTs and indicated that the area under the curve (AUC) values of hsa_circ_0008309 and hsa_circ_001242 were 0.764 and 0.784, respectively. These results suggested that hsa_circ_0008309 and hsa_circ_001242 could serve as potential diagnostic biomarkers for OSCC [139]. However, hsa_circ_0109291 was overexpressed in OSCC, which was discovered by high-throughput sequencing and then validated with qRT-PCR. In addition, the increased expression levels of hsa_circ_0109291 were associated with high TNM stage and poor overall survival of OSCC patients, suggesting the potential of hsa_circ_0109291 as a prognostic biomarker [140].

Salivary miRNAs and lncRNAs could serve as biomarkers for OSCC and other HNCs [141–143], and thus, whether the circRNAs in saliva [39] could serve as biomarkers has attracted interest. Recently, Zhao et al. found that 32 circRNAs were differentially expressed in the saliva of OSCC patients and age- and sex-matched healthy subjects. The increased level of hsa_circ_0001874 was closely associated with TNM stage and tumor grade, and the level of hsa_circ_0001971 was associated with TNM stage. In a comparison with healthy controls, ROC curve analysis showed that the AUC of hsa_circ_0001874 and hsa_circ_0001971 was 0.863 and 0.845, respectively. Moreover, the AUC for the combination of hsa_circ_0001874 and hsa_circ_0001971 reached up to 0.922, suggesting their potential as diagnostic biomarkers for OSCC. This combination could also distinguish OSCC from oral leukoplakia (OLK) with an AUC of 0.895. After surgery, the expression levels of salivary hsa_circ_0001874 and hsa_circ_0001971 decreased to levels that showed no significant difference from those of normal controls. Therefore, the authors concluded that salivary hsa_circ_0001874 and hsa_circ_0001971 could be biomarkers with high sensitivity and specificity for the early diagnosis of OSCC [144].

For laryngeal squamous cell carcinoma (LSCC), research on circRNAs was first conducted in 2016 by Xuan et al. These researchers analyzed differentially expressed circRNAs in 5 pairs of LSCC tissues and ANTs using microarray assays [145]. The upregulated circRNA and the downregulated circRNA with the highest fold-changes were hsa_circRNA_100855 and hsa_circRNA_104912, respectively. And LSCC with higher T stage, neck lymph nodal metastasis or clinical stage of LSCC exhibited higher levels of hsa_circRNA_100855 and lower levels of hsa_circRNA_104912. In addition, low hsa_circRNA_104912 expression was associated with poor differentiation [145]. As potential biomarkers for the diagnosis and prognosis of LSCC, has_circRNA_100855 and hsa_circRNA_104912 in LSCC should be further investigated to elucidate their underlying mechanisms.

The expression levels of circHIPK3 (hsa_circ_0000284) were upregulated in nasopharyngeal carcinoma (NPC) tissues compared with the ANTs, and high levels of circHIPK3 were associated with advanced clinical stage, distant metastasis, poor overall survival rate and distant metastasis-free survival (DMFS) rate in NPC patients, suggesting that circHIPK3 could serve as a prognostic marker [146]. The research conducted by Shuai et al. suggested that has_circ_0000285, another circRNA generated from the HIPK3 gene locus, was also overexpressed in NPC tissues compared to ANTs and in the serums from NPC patients compared to those from healthy controls [147]. The levels of has_circ_0000285 in the serums of NPC patients were positively associated with tumor size, TNM stage, distant metastasis and lymph node metastasis and negatively associated with the differentiation and overall survival of NPC. The serum level of has_circ_0000285 in radiation-resistant NPC was approximately three times that in radiation-sensitive NPC [147]. Above all, has_circ_0000285 could serve as a biomarker for prognosis and the efficiency of radiotherapy for NPC.

### The functions of dysregulated circRNAs in HNCs

CircPVT1 has been reported as an oncogenic circRNA in HNSCC [137]. Silencing circPVT1 decreased the proliferation and inhibited the cell cycle of the CAL27, Detroit 562 and FaDu cell lines, while also increasing the cisplatin sensitivity of Detroit 562 cells. The mut-p53-associated miR-497-5p could be specifically and directly regulated by circPVT1, and overexpression of miR-497-5p could imitate the effects of circPVT1 silencing on CAL27 cells. In the end, the cell proliferation-associated genes aurka, mki67, and bub1 were shown to function downstream of the circPVT1/miR-497-5p axis [137].

The regulatory mechanisms of circPVT1 biogenesis were also investigated in detail. Knocking down mut-p53 repressed the expression of circPVT1 through mediating the mut-p53/YAP/TEAD complex, which promotes the expression of circPVT1 at the transcriptional level. Further RNA immunoprecipitation (RIP) assays indicated that mut-p53 could stabilize the YAP and circPVT1 complexes, suggesting that circPVT1 might play a role in the regulation of itself. This hypothesis was proven by the fact that upregulated circPVT1 could facilitate the expression of circPVT1 and inhibit the expression of PVT1 [137].

However, many more studies have focused on the cancers formed at various sites in the head and neck region. This is because HNCs are relatively heterogeneous diseases that occur in complex anatomical structures, and different etiological factors and pathological and biological molecular changes are responsible for different subtypes of HNCs [148, 149]. For example, the loss of expression of common fragile site genes [150] and methylation of tumor-related genes [151] presented site-specificity in different subtypes of HNCs. Given the differentially expressed miRNAs in HNCs located at various places [152] and the tissue-specificity of circRNAs, the circRNAs in HNCs may be differentially dysregulated according to the site of the primary tumor (Table 4).

**Table 4:** The potential function and the mechanism of the dysregulated circRNAs in HNCs

CircRNAs	Chromosome	Gene symbol	Primary sites of cancer	Expression change	Functions	Possible mechanism	Reference
circPVT1	chr8	*PVT1*	HNSCC	Up	Promote proliferation and cell cycle; increase the cisplatin resistance	miRNA sponges (circPVT1/miR-497-5p/aurka, mki67, and bub1 axis)	[137]
hsa_circ_0109291	chr19	*ZNF714*	OSCC	Up	Promote proliferation and migration, inhibit apoptosis	miRNA sponges*	[140]
hsa_circ_0000284 (circHIPK3)	chr11	*HIPK3*	OSCC	Up	Promote proliferation	miRNA sponges (circHIPK3/miR-124 axis)	[155]
hsa_circ_0008309	chr2	*CUL3*	OSCC	Down	–	miRNA sponges (hsa_circ_0008309/miR-136-5p/miR-382-5p/ATXN1)	[138]
hsa_circ_0007059	chr16	*ZNF720*	OSCC	Down	Suppress proliferation, inhibit migration and invasion, promotes apoptosis	miRNA sponges (hsa_circ_0007059/AKT/mTOR pathway)	[158]
hsa_circ_0036186 (circRNA_036186)	chr15	*PKM2*	OSCC	Up	–	miRNA sponges (circRNA_036186/miR-193b-3p/ζ polypeptide axis)*	[161]
circRNA_100290	chr1	*SLC30A7*	OSCC	Up	Promote proliferation and cell cycle	miRNA sponges (circRNA_100290/miR-29/CKD6 axis)	[162]
hsa_circ_100721 (circDOCK1)	chr10	*DOCK1*	OSCC	Up	Inhibit apoptosis	miRNA sponges (circDOCK1/miR-196a-5p/BIRC3 axis)	[163]
hsa_circ:chr20:31876585–31,897,648	chr20	*BPIFB1*	LSCC	Down	–	miRNA sponges*	[171]
hg_circ_0005033	chr7	*HIBADH*	LSCC	Up	Increase the proliferation, migration, and invasion and suppress the chemotherapy sensitivity of LSCC stem cells	miRNA sponges (hg19_circ_0005033/miR-4521)	[179]
hsa_circ_0058106	chr2	*FN1*	HSCC	Up	–	miRNA sponges*	[180]
hsa_circ_0058107	chr2	*FN1*	HSCC	Up	–	miRNA sponges*	[180]
hsa_circ_0024108	chr11	*MMP1*	HSCC	Up	–	miRNA sponges*	[180]
hsa_circ_0036722	chr15	*RHCG*	HSCC	Down	–	miRNA sponges*	[180]
hsa_circ_0002260	chr5	*PAPD4*	HSCC	Down	–	miRNA sponges*	[180]
hsa_circ_0001189	chr21	*MORC3*	HSCC	Down	–	miRNA sponges*	[180]
hsa_circ_0008287	chr19	*GPATCH1*	HSCC	Down	ErbB and Hippo signaling pathways*	miRNA sponges (hsa_circ_0008287/miR-548c-3p/ErbB and Hippo pathway genes)*	[181]
hsa_circ_0005027	chr11	*ARHGAP32*	HSCC	Down	ErbB and Hippo signaling pathways*	miRNA sponges (hsa_circ_0005027/miR-548c-4p/ErbB and Hippo pathway genes)*	[181]
hsa_circ_0000284 (circHIPK3)	chr11	*HIPK3*	NPC	Up	Promote proliferation, migration, invasion	miRNA sponges (circHIPK3/miR-4288/ELF3 axis)	[146]

Note: *HNSCC* head and neck squamous cell carcinoma, *OSCC* oral squamous cell carcinoma, *LSCC* laryngeal squamous cell carcinoma, *HSCC* hypopharyngeal squamous cell carcinoma, *NPC* nasopharyngeal carcinoma, “-” means not investigated in the paper, “*” means based on bioinformatics analysis but not validated experimentally

#### CircRNAs in OSCC

OSCC is the most commonly occurring malignancy in the oral cavity, ranking ninth in cancer incidence worldwide [153]. The roles of ncRNAs in oral cancer have been studied intensively, and these molecules could serve as diagnostic biomarkers [154]. The potential circRNA biomarkers for OSCC were discussed in the previous section. CircRNAs also participated in the pathophysiological processes in the occurrence and development of OSCC. As a potential prognostic biomarker for OSCC, hsa_circ_0109291 was upregulated in OSCC [140]. After hsa_circ_0109291 expression was inhibited, the migration and proliferation were suppressed, but apoptosis was induced [140]. Similarly, Wang et al. demonstrated that circHIPK3 was overexpressed in OSCC tissues compared to ANTs and that the levels of circHIPK3 were closely associated with TNM stage and tumor grades [155]. The levels of circHIPK3 were higher in OSCC cell lines than in hNOK cell lines. Additionally, knocking down the expression of circHIPK3 inhibited the proliferation of OSCC cells, which could be partly reversed by inhibiting miR-124, suggesting that circHIPK3 may play a role in the development of OSCC via the regulation of miR-124 [155].

Li et al. predicted that hsa_circ_0008309 could combine with miR-1290, miR-136-5p, and miR-382-5p to regulate the expression of ATXN1 in OSCC by bioinformatics analysis. After the transfection of the hsa_circ_0008309 overexpression vector, the expression of hsa_circ_0008309 was upregulated, while miR-136-5p and miR-382-5p were downregulated. Then, ATXN1 overexpression was verified by western blot analysis, suggesting the role of the hsa_circ_0008309/miR-136-5p/miR-382-5p/ATXN1 pathway in OSCC [138]. Given the role of ATXN1 in Notch signaling and the EMT process [156, 157], hsa_circ_0008309 might be important for the development and progression of OSCC. At the same time, hsa_circ_0007059 was found to be downregulated in OSCC by the same research team and was significantly associated with lymph node metastasis in OSCC patients [158]. The introduction of synthetic hsa_circ_0007059 suppressed the proliferation, migration and invasion but accelerated the apoptosis of OSCC cells. The phosphorylated forms of p-AKT and p-mTOR were verified to be regulated by the expression of hsa_circ_0007059, suggesting that hsa_circ_0007059 may function through the AKT/mTOR axis in OSCC [158]. Given the oncogenic roles of the axis and its significance in the radioresistance of OSCC, hsa_circ_0007059 is a promising therapeutic target for OSCC [159, 160].

In a microarray assay, the differentially expressed circRNAs and mRNAs were identified in 5 pairs of OSCC tissues and ANTs [161]. Based on the differentially expressed circRNAs, the probable ceRNA network was constructed with bioinformatics analysis. Then, miRNAs associated with tumor progression and patient survival were screened, and those miRNAs whose target mRNAs overlapping with the differentially expressed mRNAs were selected to further refine the ceRNA network. After analysis of the miRNA-mRNA axes, the circRNA_036186/miR-193b-3p/ζ polypeptide (14–3-3ζ) axes were suggested to play a role in the development and progression of OSCCs [161]. However, more convincing functional experiments need to be performed in the future.

Compared to non-cancerous matched tissues, OSCC tissues showed upregulated circRNA_100290 by circRNA microarray and qRT-PCR analyses [162]. Knocking down circRNA_100290 induced G1/S arrest in the SCC9 cell line and inhibited the proliferation of the SCC9 and CAL27 cell lines in vitro and HN4 cells in vivo, which was mediated by downregulation of CKD6, a cyclin-dependent kinase that drives the cell cycle [162]. These effects could be neutralized by the inhibition of miR-29. The direct interaction between miR-29 and circRNA_100290 or CKD6 was demonstrated with luciferase reporter assays and EGFP/RFP reporter assays, respectively. Thus, circRNA_100290 could target CKD6 to control the cell cycle and proliferation of OSCC via sponging the miR-29 families [162].

By stimulating CAL-27 cells with human TNF-α for 48 h, an apoptotic model of OSCC was built [163]. Then, circRNA profiles and qRT-PCR verified the downregulation of circDOCK1 (hsa_circ_100721) in the apoptosis group. However, circDOCK1 levels in OSCC cell lines were higher than those in hNOK. Knocking down circDOCK1 increased the apoptosis rate in OSCC cell lines, while upregulating miR-196a-5p and downregulating BIRC3. Furthermore, miR-196a-5p mimics decreased the expression levels of both circDOCK1 and BIRC3, increasing the apoptosis rate. In OSCC tissues, circDOCK1 and BIRC3 were upregulated compared with those in ANTs, while miR-196a-5p was downregulated. Hence, circDOCK1/miR-196a-5p/BIRC3 played a vital role in the apoptosis of OSCC cells, especially during late apoptosis [163].

#### CircRNAs in LSCC

While the incidence of laryngeal cancer has decreased, the overall survival has not increased but rather decreased from 66 to 63% during the past four decades [164, 165]. These results could be ascribed to the fact that over half of patients were diagnosed with advanced cancer (stage III or IV); thus, early diagnosis is valuable for the treatments of laryngeal cancer [164]. Accumulating evidence suggests that ncRNAs play vital roles in the development of LSCC, which is the most common pathological type of laryngeal cancer [166], and could serve as diagnostic biomarkers. Evidence has shown that both miRNAs and lncRNAs were involved in LSCC [167–170], while studies on the circRNA involved in LSCC are rare.

Recently, NGS was conducted to investigate the circRNA profiles in LSCC, which could account for the circRNAs that are not present on the microarray [171]. Three moderately differentiated LSCC samples, two well-differentiated LSCC samples and five corresponding ANT samples were included. In all, more than 20 thousand circRNAs were detected, most of which were ecircRNAs. After integrating the comparison results of “moderately differentiated LSCC *vs* ANTs” and “well differentiated LSCC *vs* ANTs”, there were 18 consistently downregulated circRNAs and 5 upregulated circRNAs in LSCC. Moreover, the downregulation of hsa_circ:chr20:31876585–31,897,648 with most predicted target miRNAs was validated by qRT-PCR, demonstrating its potential as a diagnostic biomarker for LSCC [171]. However, the results need to be verified in a larger group because the sample size of this study was small, and the dysregulated circRNAs with the largest change-fold were not discussed.

Cancer stem cells are regarded as the underlying initiator of malignant tumors [172]. CD133^+^ cancer stem cells [173–176] and side populations with stem cell-like properties [177, 178] of LSCC have been isolated and intensively studied for a long period. Recently, with magnetic-activated cell sorting (MACS), CD133^+^CD44^+^ stem cells (TDP) and CD133^−^CD44^−^ non-stem cells (TDN) were successfully isolated from LSCC TU-177 cells [179]. Then, whole-transcriptome sequencing analyses (including circRNAs, lncRNAs, miRNAs and mRNAs) of TDP, TDN and parental cells (TPT) were performed. Based on the ceRNA hypothesis, the circRNA/miRNA/mRNA regulatory network was constructed in which the mRNAs were enriched in various processes and pathways of cancer progression, such as cell-cell adhesion, cell migration, double-strand break repair, and pathways in cancer. Hg19_circ_0005033 was significantly upregulated in TDP cells, and knocking down hg19_circ_0005033 suppressed proliferation, migration, and invasion and increased the chemotherapy sensitivity of TDP cells. The direct binding between miR-4521 and hg19_circ_0005033 was confirmed by a luciferase reporter assay. In addition, exogenous miR-4521 mimics could decrease the levels of hg19_circ_0005033 in TDP cells; otherwise, miR-4521 inhibition could increase the expression of hg19_circ_0005033. The upregulation of miR-4521 could be achieved by knocking down hg19_circ_0005033. Therefore, hg19_circ_0005033 might function by sponging miR-4521 to regulate the biological behaviors of LSCC stem cells [179]. However, the downstream mRNAs should be further validated, and rescue experiments should be performed to elaborate the regulatory network in LSCC stem cells.

#### CircRNAs in hypopharyngeal squamous cell carcinoma (HSCC)

HSCC is one of the most aggressive HNCs. Microarray analysis showed 2392 dysregulated circRNAs in HSCC tissues compared with ANTs [180]. Among them, hsa_circ_0058106, hsa_circ_0058107 and hsa_circ_0024108 were demonstrated to show higher expression, while hsa_circ_0036722, hsa_circ_0002260, and hsa_circ_0001189 showed lower expression in tumors than in ANTs. Then, the circRNA/miRNA/mRNA network of the above six circRNAs was constructed based on bioinformatics analysis. KEGG analysis showed that the MAPK signaling pathway and endocytosis were enriched for all 3 upregulated circRNAs. Meanwhile, the 3 downregulated circRNAs were involved in proteoglycans in cancer, choline metabolism in cancer, Wnt signaling pathway and AMPK signaling pathway [180]. Although the downstream miRNAs were estimated by the authors, the authentic functional mechanisms of altered circRNAs need to be studied further in the future.

Another study focusing on the dysregulated circRNAs in HSCC indicated that 71 circRNAs were upregulated and 102 were downregulated in tumors compared with ANTs [181]. The potential circRNA-miRNA code network [182] was predicted to unveil the functions of dysregulated circRNAs. The miRNAs targeted by the circRNAs were mainly involved in the ErbB, Hippo, Ras and Wnt signaling pathways. For further analysis of the related circRNAs in the ErbB and Hippo pathways, two subnetworks centered on miR-548c-3p were filtered out from the whole ceRNA network. Two downregulated circRNAs, namely, hsa_circ_0008287 and hsa_circ_0005027, were found to target miR-548c-3p to control the ErbB pathway genes and Hippo pathway genes that were regulated by miR-548c-3p [181]. The clinical importance of miR-548c-3p was proven by its negative correlation with the overall survival of patients with upper aerodigestive tract cancer, which was in accordance with the protective roles of hsa_circ_0008287 and hsa_circ_0005027 indicated by their lower expression level in the HSCC tissues compared to that of ANTs.

#### CircRNAs in NPC

The number of NPC patients is highest in Asia worldwide. With the modification of lifestyles and the development of radiotherapy, molecular-targeted therapies and immunotherapy, the incidence and mortality have decreased in recent years [148]. The underlying roles of circRNAs in NPC have been studied.

CircHIPK3 (hsa_circ_0000284) was overexpressed in NPC. Silencing circHIPK3 could suppress the cell proliferation, migration, and invasion of NPC cell lines, which could be neutralized by inhibiting miR-4288. ELF3 expression in NPC cells could be downregulated with the ectopic expression of miR-4288. Furthermore, knocking down circHIPK3 could inhibit the development and metastasis of NPC in vivo, inducing upregulated miR-4288 and downregulated EIF3 in xenograft tumors. Further rescue functions confirmed that circHIPK3 could promote NPC progression by the miR-4288-ELF3 axis [146]. Thus, circHIPK3 could not only act as a biomarker for prognosis but could also serve as a breakthrough point for novel therapy in NPC patients.

Epstein-Barr virus (EBV) is an etiological factor for NPC [148]. Levels of plasma EBV DNA have been shown to be prognostic biomarkers for NPC and could serve as stratification indicators of patients for treatment intensification [148]. A recent study showed that EBV could produce various circRNAs, in which expression levels of some were nearly equal to the levels of circRNAs in cells [183, 184]. These high expression levels indicated that circRNAs originating from EBV were important to the pathological process associated with EBV. Among the over 30 candidates of unique EBV circRNAs, two circRNAs generated from the RPMS1 locus, circular RPMS1_E4_E3a and circular RPMS1_E4_E2, were detected in two EBV-positive stomach tumor samples, suggesting their potential role in the cancer environment [184]. Studies have suggested that circular RPMS1_E4_E2 (named ebv-circRPMS1 in Huang et al.’s work [185] and circBART_2.2 in Toptan et al.’s work [183]) is located in both the cytoplasm and nuclei of EBV-infected NPC cell lines, including the C666–1 cell line [185] and HK1^EBV^ cells [183]. Circular RPMS1_E4_E2 was also shown to exist in EBV-positive NPC xenografts [183]. Considering the common “miRNA sponge” of circRNAs in the cytoplasm, the potential miRNAs targeted by circular RPMS1_E4_E2 were predicted and then validated by the downregulation of target miRNAs after introducing the circular RPMS1_E4_E2 overexpression plasmid. Notably, exogenous circular RPMS1_E4_E2 improved the migration of cells, indicating their essential role in the progression of tumors [185]. However, the underlying mechanisms and their roles in nuclei are still unknown.

Considering the diagnostic and prognostic value of plasma EBV DNA [186, 187] and antibodies to EBV antigens [188] for NPC, the involvement of circRNAs produced by EBV in NPC and its potential clinical applications in NPC need to be investigated in the future.

## Future prospects

The emerging research on circRNAs has gradually elucidated the biogenesis, regulation and functions of circRNAs, but the integrated landscapes of circRNAs still have not been extensively studied.

The profiles and functions of various circRNAs in HNCs have been studied alike. The expression profiles of circRNAs for different HNCs have been portrayed, and most studies focused on the “sponge” function for certain circRNAs. However, some researchers have suggested that most circRNAs contain only one or two binding sites for the same miRNA; only a tiny fraction of circRNAs were enriched of MREs for certain target miRNAs, so the function of miRNA sponges might not be shared by all circRNAs [65, 83, 118]. Thus, more attention should be focused on other functions of circRNAs in HNCs in the future, such as the regulation of gene transcription, interactions with RBPs as well as being translated. Notably, the “sponge” function was usually studied by gain-of-function and loss-of-function experiments, and it is unclear whether these experiments can demonstrate the authentic functions of circRNAs [189].

CircRNAs are more stable than mRNAs and are expressed in tissue- and development-specific manners, which are advantages for the use of circRNAs as biomarkers. Additionally, circRNAs could be secreted into body fluids and exosomes in blood [33, 190]. The circRNAs in saliva have been identified as biomarkers for oral cancer [144], and more efforts to research circRNAs as potential noninvasive biomarkers for HNCs should be made to provide auxiliary diagnostic and prognostic value of circRNAs. p53 was strongly associated with HNCs [191], and p53 mutation-associated miRNAs could act as prognostic biomarkers for HNC patients [132, 192]. Thus, whether there are other circRNAs associated with p53, in addition to circPVT1 [137], that participate in the pathophysiological processes and if they could act as promising biomarkers deserve further studies.

Given their stability and distinct subcellular cytoplasmic location, circRNAs have incredible potential to act as molecular tools or therapies for various purposes, and artificial circRNAs have been engineered with diverse methods [42]. One fascinating application of circRNAs is acting as sponges to sequester oncogenic miRNAs or proteins as well as reservoirs to store and transport certain miRNAs or proteins. Recent progress in engineered circRNAs has been inspiring. According to the ceRNA theory, an artificial circRNA targeting miRNA-122, which was indispensable for the propagation of Hepatitis C Virus (HCV), was engineered [193]. In vitro and in vivo experiments confirmed that endogenous miRNA-122 could be tightly bound and sequestered by engineered circRNA [193], shedding light on the potential of artificial circRNA in molecular medicine for hepatocellular carcinoma [194]. Similarly, an artificial circRNA named scRNA21 targeting oncogenic miR-21 was synthesized, and transfection with scRNA21 could suppress the proliferation of gastric carcinoma cells and promote apoptosis [195]. Notably, the suppression was more efficient for scRNA21 than the common miR-21 inhibitor, indicating that scRNA21 could serve as a potential effective therapeutic [195]. Therefore, synthesized circRNAs targeting oncogenic miRNAs in HNCs should be engineered to realize their translational therapeutic value.

As an increasing number of circRNAs have been shown to be translated, the transfection of artificial circRNAs that produce specific therapeutic proteins into cancer cells is another fascinating research direction [196]. Different technologies have been developed to facilitate the translation of artificial circRNAs in eukaryotic cells [197–200]. Additionally, fabricated circRNAs containing an internal ribosome entry site (IRES) could be translated in vitro as early as in 1995 [201]. Recently, the expression and translation of AAV-based artificial circRNAs based on the inserted IRES in vivo, even in a tissue-dependent manner, were realized by Meganck et al. [202]. Considering the stability of the circRNAs, the introduction of exogenous circRNAs capable of encoding proteins could allow the stable expression of certain proteins, which is important in clinical practice.

CircRNAs could be produced from EBVs and were shown to function in tumorigenesis associated with EBVs [183, 184]. Considering the role of EBVs and human papillomaviruses (HPVs) in HNCs, the circRNAs generated from these viruses and their roles in HNCs should be brought to the forefront and deserve more attention.

As discussed above, circHIPK3 was suggested to be upregulated in both OSCC and NPC, but the verified downstream miRNAs were different in the two types of cancers [146, 155]. These results indicate that there were common characteristics and distinct features between the two cancers. However, we could not exclude the possibility that circHIPK3 targeted both miRNAs in the two types of cancers nor could we rule out the possibility that circHIPK3 was upregulated in other subtypes of HNCs. Despite these limitations, the results of these reviewed studies should be applied to the same subtype of HNCs to avoid probable misapplications, even if the cancers included here were all generated from the aerodigestive tract.

Therefore, there are many unknown questions about circRNAs that need to be explored. The underlying network of circRNAs/miRNAs/mRNAs and circRNAs/RBPs and other functions of circRNAs in HNCs need to be uncovered in the future. Full elucidation of the global ceRNA and RNA/protein crosstalk under pathophysiological conditions in HNCs has exciting implications for the development of promising therapeutic approaches related to circRNAs.

## Abbreviations

ADAR1: Adenosine deaminases that act on RNA 1
ANTs: Adjacent-normal tissues
AUC: Area under curve
Cdr1as: Antisense to the cerebellar degeneration-related protein 1 transcript
CEA: Carcinoembryonic antigen
ceRNA: Competing endogenous RNA
ciRNAs: Intronic circRNAs
DCM: Dilated cardiomyopathy
DHX9: DExH-box helicase 9
DMFS: Distant metastasis-free survival
dsRNA: Double-strand RNA
EBV: Epstein-Barr virus
ecircRNAs: Exonic circRNAs
EIciRNAs: Exon-intron circRNAs
EMT: Epithelial-mesenchymal transition
f-circRNAs: Fusion circRNAs
FISH: Fluorescence in situ hybridization
HNCs: Head and neck cancers
hnRNPs: Heterogeneous nuclear ribonucleoprotein
HNSCCs: Head and neck squamous cell carcinomas
HPV: Human Papillomavirus
HSCC: Hypopharyngeal squamous cell carcinoma
IRES: Internal ribosome entry site
LDH: Lactate dehydrogenase
lncRNA: Long ncRNA
LNM: Lymph node metastasis
LSCC: Laryngeal squamous cell carcinoma
MACS: Magnetic-activated cell sorting
Mbl: Muscleblind
miRNA: microRNA
MREs: miRNA response elements
ncRNA: non-coding RNA
NF90/NF110: Nuclear factor 90/110
NGS: Next-generation sequencing
NPC: Nasopharyngeal carcinoma
ORFs: Open reading frames
OSCC: Oral squamous cell carcinoma
QKI: Quaking
qRT-PCR: Real-time quantitative reverse transcription-polymerase chain reaction
RBM20: RNA-binding motif protein 20
RBPs: RNA binding proteins
RIP: RNA immunoprecipitation
ROC: Receiver operating characteristic
snRNP: Small nuclear ribonucleoprotein
SR: Serine–arginine
